The article "Melatonin Attenuates Cisplatin-Induced Ototoxicity via Regulating the Cell Apoptosis of the Inner Ear" was retracted in 2023. Reasons: signs of a paper mill; compromised peer review; unreliable results or conclusions.

# Melatonin Attenuates Cisplatin-Induced Ototoxicity via Regulating the Cell Apoptosis of the Inner Ear

**DOI:** 10.1155/2022/7160816

**Published:** 2022-09-01

**Authors:** Na Wang, Anting Xu, Hao Zhang, Yongju Zhang, Rongcui Sui, Xintai Fan, Lingxiao Hou, Li Shi

**Affiliations:** ^1^Department of Otolaryngology and NHC Key Laboratory of Otorhinolaryngology, The Second Hospital of Shandong University, Jinan 250033, Shandong Province, China; ^2^Department of Otolaryngology, Jinan Children's Hospital, Jinan 250022, Shandong Province, China

## Abstract

**Objective:**

The mechanism of ototoxicity caused by cisplatin is currently unclear, and the induced apoptosis may play an important role in inner ear injury. Melatonin has high antioxidant and antiapoptotic effects. This study is aimed at clarifying the protective effect on the inner ear and the underlying mechanism of melatonin.

**Design:**

The mice and HEI-OC1 cells were randomly separated into four groups: control group, cisplatin group, melatonin group, and cisplatin exposure after melatonin pretreatment group. *Place and Duration of the Study.* From September 2018 to September 2021, all experiments were completed at the Second Hospital of Shandong University. And the study was approved by the Ethics Committee of the Second Hospital of Shandong University (KYLL-2020 (KJ) A-0191). *Methodology.* Mice were pretreated with peritoneal injection of melatonin prior to the application of cisplatin. Auditory Brainstem Response (ABR) test was performed before and after treatment, then the temporal bones were collected for histology investigation. HEI-OC1 cells were pretreated with melatonin before adding cisplatin. The apoptosis of HEI-OC1 cells was observed by MTS, TUNEL, and flow cytometry, respectively. Moreover, the mRNA expression of apoptosis-related factors was detected by qRT-PCR.

**Results:**

ABR and morphological analysis showed that cisplatin caused damage to the function and structure of the inner ear. MTS, TUNEL, and flow cytometry showed that the application of cisplatin caused a significant increase in the apoptosis level of HEI-OC1 cells, and melatonin pretreatment reduced this damage. Moreover, melatonin pretreatment reversed the mRNA expression changes of apoptosis-related factors induced by cisplatin.

**Conclusions:**

Apoptosis is involved in the inner ear dysfunction caused by cisplatin. Melatonin reduces the ototoxicity of cisplatin by regulating the induced apoptosis response.

## 1. Introduction

Cisplatin (DDP) is a chemotherapeutic drug which is commonly used in clinical practice to treat solid tumors such as ovarian and testicular carcinoma, cervical carcinoma, lung carcinoma, and squamous head and neck carcinoma. However, severe dose-limiting side effects such as ototoxicity, neurotoxicity, nephrotoxicity, and myelotoxicity may occur during cisplatin-based chemotherapy [1, 2]. Although hydration therapy and diuretics could significantly relieve nephrotoxicity, ototoxicity is still a common cause of the reduction or discontinuation of cisplatin [3]. Studies have shown that cisplatin-induced hearing loss is usually bilateral, with higher frequencies at the start and lower-frequency hearing loss over time [4]. And in the chemotherapy treatment of head and neck tumors, cisplatin can also cause hearing loss in patients [5].

Accumulated studies proved that about 40%~97% of children and 20%~60% of adults treated with cisplatin can develop ototoxicity, which was mainly characterized by bilateral irreversible sensorineural hearing loss (SNHL) and might be associated with tinnitus [6–8]. The main targets of drug action are organ of Corti [7, 9], spiral ganglion [10], and stria vascularis [11]. The damage to the organ of Corti is mainly concentrated on the outer hair cells, of which the basal turn was the most obvious at early stage. With the increase of dose, the inner hair cells may also be damaged [9–11]. Although the focus of researches was cisplatin-induced apoptosis, the mechanism of cisplatin ototoxicity is not fully understood. Studies have shown that cisplatin can cause DNA damage, mitochondrial dysfunction, and increase reactive oxygen species (ROS) production [12, 13]. ROS activates c-Jun N-terminal kinase (JNK) then transfers to the nucleus to activate genes in the cell death pathway. These products induce mitochondria to release cytochrome-c (Cyt-c), which ultimately activate a series of caspases that play a key role in the intrinsic apoptotic pathway [14, 15].

Melatonin, N-acetyl-5-methoxytryptamine, is an endogenous steroid hormone with multiple effects, which can not only directly scavenge free radicals but also indirectly regulate the activity and expression of various endogenous antioxidant enzymes. In addition, it also can protect mitochondrial function, reduce the leakage of electrons in the respiratory chain and the increase of ROS, and inhibit the vicious circle of increased ROS [16, 17]. Since melatonin has high fat solubility and low plasma protein binding rate, it can easily pass through the blood-brain barrier to regulate multiple physiological activities. Studies have shown that melatonin can reduce oxidative stress, apoptosis, and inflammation and regulate mitochondrial function and sex hormones in germ cells, improving reproductive damage and function during chemotherapy [18]. In addition, melatonin can also prevent kidney damage [19], ovarian damage [20], and neurodegeneration during chemotherapy [21]. It has been proved that the antioxidant effect of melatonin can reduce the toxic effects of cisplatin and promote the efficacy of cancer therapy [22, 23].

In the present study, the effects of melatonin pretreatment on the auditory dysfunction and inner ear morphological changes caused by cisplatin were investigated. Moreover, the mRNA expression levels of apoptosis-associated factors Bax, caspase-3, caspase-9, and Bcl-2 were checked. This study was aimed at exploring the effects of melatonin on the auditory dysfunction and inner ear morphological changes caused by cisplatin and its mechanism.

## 2. Materials and Methods

### 2.1. Cell Culture and Treatment

House Ear Institute-Organ of Corti 1 (HEI-OC1) cell line was derived from the organ of Corti of the transgenic mouse Immortomouse™ and cultured in high-glucose Dulbecco's modified Eagle's medium (DMEM) supplemented with 10% fetal bovine serum (FBS), 100 *μ*g/ml streptomycin, and 100 U/ml penicillin. Then, the cells were incubated at 33°C in a humidified incubator with 5% carbon dioxide (CO_2_). HEI-OC1 cell line is an auditory hair cell line that expresses specific markers of auditory hair cells on the surface of HEI-OC1 cells, and the cells are sensitive to ototoxic drugs [24]. It is a very useful model to investigate mechanisms of action of ototoxic chemicals.

The cultured cells were divided into 4 groups: control group, cisplatin-treated group, melatonin-treated group, and melatonin-pretreated cisplatin group. The cell treatment process was as follows: the control group was treated with the same amount of reagent buffer; the cisplatin-treated group was treated with cisplatin for 24 hours; the melatonin-treated group was treated with melatonin for 2 hours and then replaced with fresh medium; and the melatonin-pretreated cisplatin group was treated with cisplatin for 24 hours after 2 hours of melatonin pretreatment. Cisplatin was used at a concentration of 10 *μ*g/ml and melatonin at a concentration of 5 *μ*mol/ml.

### 2.2. The Establishment of Animal Models

A total of 24 C57BL/6 mice aged at one month old and weighed between 20 and 25 g were fed in an ideal laboratory conditions, with 12 h light and 12 h darkness cycles, and with free access to food and water. The experimental protocol was approved by the Ethics Committee of the Second Hospital of Shandong University (permit number: KYLL-2020 (KJ) A-0191). All mice with the outer or middle ear infections were excluded from the experiment. The mice were anesthetized by intraperitoneal injection of pentobarbital sodium at a dose of 100 mg/kg according to the body weight. Then, the mice were randomly separated into four groups: control group, cisplatin group, melatonin group, and cisplatin exposure after melatonin pretreatment group. Mice injected intraperitoneally with normal saline served as the control group, while the mice in the cisplatin group, melatonin group, and cisplatin exposure after melatonin pretreatment group were severally intraperitoneally injected with cisplatin (Sigma, Alexandria, VA, USA) (8 mg/kg), melatonin (Sigma, Alexandria, VA, USA) (10 mg/kg), and melatonin (10 mg/kg)+cisplatin (8 mg/kg). Among them the melatonin and cisplatin injections should be separated by two hours in the cisplatin exposure after melatonin pretreatment group. Four groups of mice were reinjected two days after the first medication. An initial Auditory Brainstem Response (ABR) test was performed before treatment. One month after the first injection, a new ABR was performed. Temporal bones were collected for histology investigation.

### 2.3. MTS Assay

3-(4,5-Dimethylthiazol-2-yl)-5-(3-carboxymethoxyphenyl)-2-(4-sulfophenyl)-2H-tetrazolium (MTS) assay was performed to determine the toxicity of potential drugs and toxicants to cells. HEI-OC1 cells were seeded in a 96-well plate at a density of 1 × 10^4^ cells per well. Cell grouping and drug treatment were described above. Subsequently, the cell culture medium was discarded and replaced by the DMEM with fresh 5% FBS and 200 *μ*l per well along with 20 *μ*l MTS reagent and then cultured for another 4 hours at 33°C with 5% CO_2_. Finally, the OD_490nm_ value of each group was measured using a microplate reader (Stat FAX 2100; Los Angeles, CA, USA). The experiment was repeated three times, with four replicates in each group.

### 2.4. qRT-PCR

Total RNA of HEI-OC1 cells in each group and the cochlea of each group of mice were extracted by TRIzol reagent (Invitrogen, Carlsbad, CA, USA), and the extracted RNA concentration and quality were measured by NanoDrop spectrophotometer (Thermo Fisher Scientific, Waltham, MA, USA). Then, complementary DNA (cDNA) was synthesized using a SuperScript™ III First-Strand Synthesis SuperMix (Invitrogen, Carlsbad, CA, USA) for qRT-PCR. The qRT-PCR reactions were performed by a StepOne™ Real-Time PCR System (Applied Biosystems, Foster City, CA, USA) using the following five primer pairs: Bcl-2: forward: 5′-ACTTCTCTCGTCGCTACCGTC-3′, reverse: 5′-CCCCATCCCTGAAGAGTTCCT-3′; Bax: forward: 5′-AGGGTTTCATCCAGGATCGAGCA-3′, reverse: 5′-CAGCTTCTTGGTGGA-CGCATC-3′; caspase-3: forward: 5′-GAAACACTGGAAGCACGGAT-3′, reverse: 5′-CAAGGTCAGAATGCA-CCAGA-3′; caspase-9: forward: 5′-AGCACCTGGTTACTATTCCTG-3′, reverse: 5′-TAAATTCTAGCTTGT-GCGCGTA-3′; and *β*-actin: forward: 5′-CACCATCGCCAGGACCAT-3′, reverse: 5′-GAACTCCTCGGGACCCAG-3′.

The program operating conditions of qRT-PCR were 95°C, 5 min; 95°C, 10 s, 60°C, 30 s, 72°C, 20 s, 40 cycles; 72°C, 5 min, and finally kept at 4°C. The 2 − ΔΔCT method was used to calculate the relative expression of genes.

### 2.5. TUNEL Assay

Terminal Deoxynucleotidyl Transferase mediated dUTP Nick End Labeling (TUNEL) assay was used to detect the nuclear DNA fragmentation of tissue cells during the late stage of apoptosis, which was performed using the TUNEL Apoptosis Detection Kit (Yeasen Biotech Co, Shanghai, China) according to the manufacturer's protocol. Subsequently, images were acquired using a fluorescence microscope (Leica DM3000, Germany) and analyzed with ImageJ software.

### 2.6. Flow Cytometry

The cell culture fluid was carefully collected into a centrifuge tube and digested using Ethylenediaminetetraacetic acid- (EDTA-) free trypsin until the cells could be gently blown down with a pipette. Then, the previous cell culture solution was collected and all adherent cells were blown down and apart. Next, the cells were centrifuged at about 1000 rpm for 5 min and the supernatant was extracted. Approximately 1 ml of 4°C prechilled PBS was used to resuspend the cells. After being centrifuged, the supernatant was discarded. The flow cytometry was performed using the Annexin V-FITC/PI Apoptosis Detection Kit (4A Biotech, Beijing, China) according to the manufacturer's protocol. In detail, the binding buffer was diluted by deionized water (4 ml 4× binding buffer+12 ml deionized water) and the cells were resuspended with 1× binding buffer and adjusted to a concentration of 1‐5 × 10^4^/ml. 100 *μ*l of the cell suspension and 5 *μ*l Annexin V-FITC were added into a 5 ml flow tube and mixed well, supplementing with which was incubated at room temperature for 5 minutes in the dark. After adding 10 *μ*l of 20 *μ*g/ml Propidium Iodide (PI) solution and 400 *μ*l of PBS, the flow cytometry was performed immediately using a BD Accuri C6 flow cytometer (BD Bioscience, USA).

### 2.7. ABR

After being successfully narcotized, the mice were put into a sound booth. The collecting electrode, reference electrode, and grounding electrode were severally inserted into the apex of the head, mastoid area, and the midline of the back of the mouse. Then, the external speaker was moved to the auricle of the mouse. Each mouse was subjected to pure tone detection in turn, and the pure tones were selected at 4 kHz, 8 kHz, 16 kHz, and 32 kHz, and the audiometry results were recorded by RZ6 MULTI-I/O PROCESSOR (Tucker Davis Technologies, Alachua, FL, USA) for statistical analysis.

### 2.8. Cochlear Anatomy

The mice were quickly sacrificed after anesthesia, after which the cranial cavity of the mouse was opened and the temporal bone was quickly removed and placed in a precooled 2.5% glutaraldehyde fixative. Then, the connective tissues around the cochlea were quickly removed under the microscope and a hole was made on the top of the cochlea, the stapes were removed, and the round window membrane was opened. 2.5% glutaraldehyde fixative was slowly injected into the small hole at the top of the cochlea with a syringe. The perfused cochlea was then placed in an EP tube containing a precooled 2.5% glutaraldehyde fixative and in a refrigerator at 4°C for at least 4 hours. Next, precooled 1% EDTA solution was used for decalcification, and the decalcification solution was changed every day for 10 days. The whole decalcification process occurred in the 4°C refrigerators.

### 2.9. Hematoxylin-Eosin (HE) Staining

The cochlear specimens in four groups were severally dehydrated and then embedded in paraffin. Specimens were cut into 4 *μ*m thick sections, dewaxed and dehydrated in gradient xylene, and stained with a hematoxylin-eosin kit according to the manufacturer's instructions. Sections were then observed and photographed using an Olympus optical microscope (Tokyo, Japan). Staining intensity was analyzed by Image-Pro Plus 6.0 software and expressed as IOD value.

### 2.10. Whole-Mount Staining

The outer layer of the decalcified mouse cochlea was removed under a dissecting microscope, and the basement membrane was peeled off from the modiolus. Then, the stria vascularis, vestibular membrane, and cover film were removed. The basement membrane was transferred to a four-well dish and added with 100 *μ*l 4% paraformaldehyde (PFA), which was fixed for 10-15 min. After that, 100 *μ*l 0.1% Triton X-100 was added and stood at room temperature for 10 min after being washed three times with PBS. Next, the Phalloidin (Sigma Aldrich, St Louis, MO, USA) diluted at 1 : 500 was added into the basement membrane for 30 min and then washed three times with PBS. Subsequently, 1 : 250 diluted DAPI (Sigma Aldrich, St Louis, MO, USA) was added into the membrane and incubated at room temperature for 10 min. The basement membrane was taken out, placed on a glass slide, and sealed with mounting medium (PBS: glycerol = 1 : 1). The image was collected with a confocal microscope (LSM700, Carl Zeiss, Germany).

### 2.11. Real-Time Cell Proliferation

To monitor the effects of cisplatin and melatonin on HEI-OC1 proliferation in real time, we used the ImageXpress Pico system combined with CellReporterXpress® imaging acquisition and analysis software for cell detection. Cell viability was detected at certain time intervals, and the results were visualized and quantitatively analyzed.

### 2.12. Statistical Analysis

The data was analyzed using SPSS 25.0 software and GraphPad prism 6.0 and presented as median ± SD. The differences between the two groups were compared by Students' *t*-test, while those among three groups or above were analyzed by chi-squared test. The difference was significant when *p* < 0.05.

## 3. Results

### 3.1. Melatonin Significantly Attenuates Cisplatin-Induced Hearing Loss

To explore the influence of melatonin on the hearing of mice, the ABR value was investigated before and after treatment in all mice. The posttreatment ABR values of the four groups were calculated and compared. The result showed that the ABR in each group had no significant difference before treatment, while that was markedly different from the control groups in other groups after treatment (Figure 1(a)). In detail, the hearing threshold of the cisplatin group at 4 kHz, 8 kHz, 16 kHz, and 32 kHz was higher than that in the control group, which was obviously reduced by melatonin. However, there were no significant differences in the melatonin group compared to the control group. These indicated that cisplatin could cause hearing loss in full frequency, whereas melatonin pretreatment could inhibit cisplatin-induced hearing loss.

### 3.2. Melatonin Protects Inner Ear Hair Cells from Cisplatin Damage

To observe the morphological changes of the Corti on the basement membrane, HE staining and phalloidin staining were conducted. HE staining showed that the inner and outer hair cells of the control group and the melatonin group had normal morphology, clear structure, and neat arrangement. Whereas, in the cisplatin group, the morphology of the hair cells was abnormal, part of the outer hair cells was missing, and the basement membrane was shrunk. Besides, there was no obvious loss of inner hair cells. Compared with the cisplatin group, the morphological change and the loss of the outer hair cells in the cisplatin exposure after melatonin pretreatment group were reduced (Figure 1(b)). Phalloidin staining showed that the outer hair cells of the cisplatin group were significantly absent, while the inner hair cells were substantially intact. Pretreatment with melatonin obviously reduced the loss of outer hair cells (Figure 1(c)). The consequence demonstrated that the pretreatment with melatonin obviously reduced the loss of outer hair cells.

### 3.3. Melatonin Protects the Viability of HEI-OC1 Cells

To investigate the influence of melatonin on the cell viability of HEI-OC1 cells, MTS analysis was performed. Compared with the control group, the cell viability of the cisplatin group was remarkably reduced (Figure 2). No significant difference was found between the control group and the melatonin group. However, the cell viability of the cisplatin exposure after melatonin pretreatment group was significantly higher than that of the cisplatin group. Hence, melatonin pretreatment could protect the activity of HEI-OC1 cells.

### 3.4. Melatonin Protects Inner Ear Hair Cells by Regulating Apoptosis

To detect the cell apoptosis of HEI-OC1 cells in four groups, TUNEL assay was conducted. Cells in the cisplatin group showed obvious cell nuclear DNA breakage during apoptosis, while the apoptotic cells in the cisplatin exposure after melatonin pretreatment group were significantly reduced (Figure 3). Flow cytometry revealed that the apoptosis rate was significantly increased in the cisplatin group, which was inhibited by melatonin (Figure 4). This also indicated that melatonin pretreatment reduced the activation of apoptosis caused by cisplatin.

To confirm that melatonin can alleviate the apoptosis of inner ear hair cells caused by cisplatin, qRT-PCR was used to detect the mRNA expression of apoptosis-related factors. Consequently, the expression levels of Bax, caspase-3, and caspase-9 were all increased, while the expression of Bcl-2 was decreased after melatonin pretreatment compared with the cisplatin group both in vivo and in vitro (Figure 5).

## 4. Discussion

With the increasing incidence of tumors and the widespread use of platinum-based chemotherapy drugs, complications such as SNHL caused by platinum-based preparations has attracted more and more attention. Cisplatin is currently the most widely used platinum drug, with strong broad-spectrum anticancer activity. The study showed that after systemic administration of cisplatin in mice, it was also detected in the perilymph of the inner ear, suggesting that it may enter the cochlear hair cells through its basolateral membrane [25]. Cisplatin-induced cochlear toxicity may also be due in part to loss of cochlear homeostasis as well as hair cell damage [26], and disruption of cochlear homeostasis can also indirectly affect hair cell survival [27]. In this study, we found that cisplatin can cause hearing loss in mice through the ABR test. The cochlea HE staining and basement membrane phalloidin staining also showed that the organ of Corti had morphological changes after applying cisplatin, further confirming that cisplatin affects the auditory function of the inner ear.

Many studies have elucidated that the cytotoxic mechanism of cisplatin includes DNA damage, ROS formation, mitochondrial dysfunction, and caspase activation [28, 29]. Cisplatin causes overproduction of ROS [30]. Moreover, the accumulated ROS can not only activate JNK and P38 MAPK but also induce mitochondria to release Cyt-c, and finally activates caspase-8, caspase-9, and caspase-3 in the intrinsic apoptotic pathway [14, 15]. Caspase-3 is a key protein in the caspase protein cascade that leads to apoptosis and may be one of the last executors of apoptosis events [31–33]. Cisplatin-induced apoptosis may be the main factor of ototoxicity. Figure 2 shows that cisplatin-induced hair cell loss and melatonin have a protective effect on cisplatin-induced hair cell damage. Whether it is the damage of cisplatin on hair cells or the protective effect of melatonin on the damage of hair cells caused by cisplatin, it is only manifested in outer hair cells. It shows that cisplatin mainly damages the hearing of mice through the regulation of oxidative stress in outer hair cells and has little effect on inner hair cells. The Bcl-2 family of proteins is the central regulator of caspase activation, and the opposition of antiapoptotic and proapoptotic factors determines cell survival [34]. Some of its members promote apoptosis, such as Bad, Bid, and Bax, while some members prevent cell apoptosis, such as Bcl-2, Bcl-x, and Bcl-w. Bcl-2 can prevent the release of Cyt-c from the mitochondria to the cytoplasm, thereby inhibiting cell apoptosis [30, 35, 36]. Bcl-2 can inhibit the expression of the proapoptotic gene Bax and the generation of free radicals. The proapoptotic mechanism of Bax is achieved by promoting the release of Cyt-c, which leads to DNA damage and apoptosis through the activation of caspase-mediated pathways [37, 38]. In this study, MTS assay showed that cisplatin significantly inhibited cell proliferation and cell viability, while TUNEL and flow cytometry exhibited that cisplatin significantly promotes the cell apoptosis. qRT-PCR indicated that caspase-3, caspase-9, and Bax were overexpressed, while Bcl-2 was decreased both in vivo and in vitro after the application of cisplatin. These results supported the hypothesis that cisplatin induces apoptosis through Bcl-2, Bax, caspase-3, and caspase-9 signaling pathways.

Cisplatin ototoxicity may be the result of multiple pathways, of which oxygen free radical damage and apoptosis are the most noticeable. Therefore, the research on the protection of ototoxicity caused by cisplatin mainly focuses on antioxidants and antiapoptotic drugs. Melatonin is one of the hormones secreted by the brain pineal gland, which is an effective endogenous free radical scavenger and participates in the antioxidant system to prevent oxidative damage to cells. In the current study, we found that the morphological changes of the inner ear caused by cisplatin were reduced, and the expression of related apoptotic factors was also abnormally expressed after pretreatment with melatonin. Moreover, melatonin pretreatment was proved to reduce hearing loss in mice and the loss of inner ear hair cells as well as regulate the expression of Bax, caspase-9, caspase-3, and Bcl-2. These results indicated that melatonin can interfere with the apoptosis signaling pathway in mitochondria to protect the ototoxicity of cisplatin to hair cells, which were in line with other studies [2, 39, 40]. Our research provides a theoretical basis for melatonin to affect neural deafness through the regulation of oxidative stress. At the same time, the clinical application of melatonin may have a driving effect on reducing the ototoxicity of other drugs, such as aminoglycosamines.

## 5. Conclusions

In summary, cisplatin damages inner ear hair cells and leads to SNHL. Cell apoptosis is involved in inner ear dysfunction caused by cisplatin. Melatonin protects ototoxicity caused by cisplatin through its antiapoptotic effect, which might be mediated by regulating Bcl-2, Bax, caspase-3, and caspase-9 apoptosis pathway in the inner ear.

## Figures and Tables

**Figure 1:** Melatonin significantly attenuates cisplatin-induced hearing loss. (a) Comparison of frequency hearing thresholds of mice in each group after cisplatin and melatonin pretreatment. The cisplatin group has significantly higher thresholds in all frequencies than the control group. Melatonin pretreatment attenuated the cisplatin-induced hearing loss. In addition, the control group and the melatonin group do not have any significant difference (∗*p* < 0.05, ∗∗*p* < 0.01). (b) Hematoxylin-eosin staining showed the Corti's morphological change of the four groups. In the cisplatin group, the outer hair cells were obviously missing, the inner hair cells had abnormal morphology, and the basement membrane became shrunk. Pretreatment of melatonin could reduce this damage (200×). (c) Basement membrane phalloidin staining showed the loss of outer hair cells after cisplatin treatment and melatonin pretreatment. The hair cells were stained using phalloidin (green), the nuclei were stained with DAPI (blue). Melatonin pretreatment can reduce hair cell loss caused by cisplatin, bar = 20 *μ*m.

**Figure 2:** Melatonin protects the viability of HEI-OC1 cells. (a) Real-time cell proliferation of the four groups. The control group (green curve), the cisplatin group (black curve), the melatonin group (brown curve), the melatonin pretreatment group (purple curve). (b) The bar graph shows quantification of the results, each value represents the average of three independent experiments. MTS assay revealed that cisplatin inhibited cell viability, and melatonin had a protective effect on cisplatin cytotoxicity, ∗∗∗*p* < 0.001.

**Figure 3:** Melatonin attenuates cisplatin-induced apoptosis in HEI-OC1 cells. (a) The morphological characteristics of HEI-OC1 cells were compared using the TUNEL assay. The green fluorescence within the nucleus represented DNA breakage. Cells in the cisplatin group display obvious apoptotic features. Fewer cells show these apoptotic characteristics in the cisplatin exposure after melatonin pretreatment group, bar = 20 *μ*m. (b) TUNEL assay showed a significant increase in the apoptosis rate of the cisplatin group. After melatonin pretreatment, the apoptosis rate decreased, ∗∗*p* < 0.01.

**Figure 4:** Melatonin reduces the proportion of apoptotic HEI-OC1 cells induced by cisplatin. Flow cytometry showed the ratio of apoptotic cells. The flow cytometry result was the same as TUNEL assay. Melatonin pretreatment reduced apoptosis caused by cisplatin cytotoxicity (∗∗∗*p* < 0.001).

**Figure 5:** Melatonin inhibits cisplatin-induced expression of apoptosis-related proteins in HEI-OC1 cells and mouse basement membrane. (a) qPCR was used to detect apoptosis-related protein expression in HEI-OC1 cells. There was no statistical difference between the control group and the melatonin group. In the cisplatin group, the mRNA expression of Bax, caspase-3, and caspase-9 increased significantly, and the mRNA expression of Bcl-2 decreased. All these changes could be mitigated by melatonin pretreatment (∗*p* < 0.05, ∗∗*p* < 0.01, ∗∗∗*p* < 0.001). (b) qPCR was used to detect apoptosis-related protein expression in mouse basement membrane. There was no statistical difference between the control group and the melatonin group. In the cisplatin group, the mRNA expression of Bax, caspase-3, and caspase-9 increased significantly, and the mRNA expression of Bcl-2 decreased. All these changes could be mitigated by melatonin pretreatment (∗*p* < 0.05, ∗∗*p* < 0.01, ∗∗∗*p* < 0.001).

## Data Availability

No data were used to support this study.
